This article has been retracted.

# Analysis of the Reactivity of Aspirin and Clopidogrel and Its Influencing Factors in Patients with Coronary Heart Disease at High Altitude

**DOI:** 10.1155/2021/2849982

**Published:** 2021-10-31

**Authors:** Rong Chang, Jinchun Wu, Xiaofei Zhang, Yi Ye, Wenqin Zhou, Yanmin Liu

**Affiliations:** ^1^Department of Cardiology, Shenzhen Longhua District Central Hospital, The Affiliated Central Hospital of Shenzhen Longhua District, Guangdong Medical University, No. 187 Guanlan Road, Longhua District, Shenzhen, Guangdong 518109, China; ^2^Department of Cardiology, Qinghai Provincial People's Hospital, Xining 810007, China

## Abstract

**Objective:**

To evaluate the efficacy of dual-antiplatelet treatment (DAPT) in patients with coronary heart disease (CHD) at high altitude by using thrombelastogram (TEG) and to analyze the related biochemical factors affecting drug reactivity.

**Methods:**

Totally 118 CHD patients who admitted to the Qinghai People's Hospital from September 2019 to September 2020 were enrolled in the group. Those people have lived in Qinghai for a long time. Seven days after DAPT, venous blood was collected on an empty stomach in the early morning of the next day; blood routine, coagulation function, and biochemical items were tested. Thrombelastogram (TEG) was used to draw curves to calculate platelet, coagulation and fibrinolysis functions, and drug inhibition rate. Patients were divided into the aspirin resistance (AR) group, clopidogrel resistance (CR) group, dual-antiplatelet drug resistance (DAR) group, and drug-sensitive group according to different inhibition rates. The drug efficacy was analyzed, and the clinical data, biochemical indexes, and TEG parameters of each group were compared to identify the risk factors of drug resistance.

**Results:**

Those 118 CHD patients at high altitude were incorporated into the study, ranging from 38 to 84 years of age, including 81 males (68.64%) and 37 females (31.36%). The platelet function and coagulation-fibrinolysis function were detected by TEG, and MA_THROMBI_, MA_ADP_, and MA_AA_ were higher than the reference range. There were 82 cases (69.49%) of drug resistance, 36 cases (32.53%) of drug sensitivity, 17 cases (14.41%) of AR alone, and 16 cases (12.71%) of CR alone. There was no significant difference in age, gender, BMI, oxygen saturation, TG, GFR, and history of diabetes and hypertension between ACS and CCS groups (*P* > 0.05). PLT and FIB in the ACS group were higher than those in the CCS group, and the difference was statistically significant (*P* < 0.05). In addition, MA_THROMBIN_, MA_FIBRIN_, E, A, A30, and coagulation composite index were also higher than those in the CCS group, with a statistically significant difference (*P* < 0.05). Univariate analysis and logistic regression analysis suggested that age, HbA1c, FBG, and diabetes were the main factors of drug resistance.

**Conclusion:**

Antiplatelet drugs aspirin and clopidogrel resistance are associated with increased age, elevated HbA1c and FBG, and diabetes. Therefore, it is necessary to take reasonable treatment measures based on the actual situation of patients.

## 1. Introduction

Along with the development of society, the incidence of cardiovascular diseases worldwide is increasing year by year, and this trend is becoming increasingly fierce among young and middle-aged people [1]. It is reported that there are 330 million people suffering from cardiovascular diseases in China, among which 11 million are coronary heart disease (CHD) [2]. Meanwhile, epidemiological data reveal that acute coronary syndrome (ACS), stroke, lower extremity arterial thrombosis, and venous thromboembolism are more likely to occur at high altitude and low pressure and hypoxia [3]. Thus, prevention and treatment of CHD is a key step to promote people's health and improve their quality of life in plateau areas.

Dual-antiplatelet treatment (DAPT) [4] can effectively prevent thrombosis, so it greatly improves the long-term prognosis of CHD and even reduces the incidence of major adverse cardiovascular events (MACEs) in patients [5]. CHD patients prevent the development or deterioration of CHD by means of DAPT [6]. Aspirin and clopidogrel [7] are still effective drugs for first-line treatment and second-line prevention of CHD patients. However, some studies have shown that, with strict DAPT treatment, some patients still have postoperative thrombosis, which may be caused by the insufficient inhibitory effect of double anti-drugs on platelets [8]. The occurrence of such incidents is related to various factors. Hence, how to accurately measure the number of platelets at high altitude, evaluate the platelet function and monitor the efficacy of antiplatelet drugs in patients, and then, explore the occurrence factors of AR and CR are relevant to the diagnosis and treatment of CHD at high altitude and the clinical application effect of antiplatelet drugs. Simultaneously, thromboelastogram (TEG) [9], as an effective way to monitor blood coagulation state, converts the mechanical characteristics of blood clot formation into electrical signals to predict complex blood coagulation state, comprehensively evaluates the influence of plasma and blood cell components on blood coagulation and fibrinolysis state, and represents the blood coagulation state of patients more realistically and systematically than traditional detection methods.

In this study, TEG was used to evaluate the DAPT effect of CHD patients at high altitude, and the causes of antiplatelet drug resistance were deeply explored. It is quite crucial to prevent the recurrence of thrombotic diseases at high altitude, reduce the mortality, formulate the optimal plan for patients, and finally, achieve the best clinical diagnosis and treatment effect.

## 2. Research Process

### 2.1. Patient Data

A total of 118 CHD patients who admitted to the Qinghai People's Hospital from September 2019 to September 2020 were enrolled in the group. Those people have lived in Qinghai for a long time, including 81 males (68.64%) and 37 females (31.36%), aged 64.9 years. Other clinical information of patients were collected, including history of smoking and clinical complications such as hypertension, type 2 diabetes, and chronic kidney disease. This study was approved by the hospital ethics committee (2019006), and the patients signed the informed consent form.

#### 2.1.1. Inclusion Criteria

① Complete clinical data
② Living in Qinghai for a long time (at least 30 years)
③ Meeting the WHO diagnostic criteria for CHD in 1979 and diagnosing as vascular lesions by coronary angiography or coronary CT [10]
④ The patient is informed and willing to cooperate

#### 2.1.2. Exclusion Criteria

① Unstable hemodynamics
② All kinds of blood diseases, hemorrhagic disorders, or bleeding tendency
③ Aspirin or clopidogrel allergy or contraindication [11]
④ Those who are currently taking platelet membrane glycoprotein receptor antagonists, other thienopyridines, and nonsteroidal anti-inflammatory drugs or receiving anticoagulants
⑤ Serious chronic diseases such as glomerular filtration rate (GFR) 60 mL/min and alanine aminotransferase (ALT) 2 times the normal upper limit
⑥ Refusing to sign the informed consent form

### 2.2. Research Process

#### 2.2.1. Diagnosis of CHD Patients

Patients who met the inclusion criteria were divided into the acute coronary syndrome (ACS) group and chronic coronary syndrome (CCS) group according to [12] the Guidelines for Rapid Diagnosis and Treatment of Acute Coronary Syndrome (2019) and Guidelines for Management of Chronic Coronary Syndrome (2019). Eventually, we included 66 with ACS (56.00%) and 52 with CCS (44.00%).

#### 2.2.2. Main Research Contents

All subjects were given aspirin enteric-coated tablets (100 mg × 30 tablets) 100 mg/d and clopidogrel hydrogen sulfate tablets (75 mg × 7 tablets, Sanofi-Aventis) 75 mg/d or aspirin 300 mg and clopidogrel 300 mg on the first day of admission; all those drugs were changed to the abovementioned conventional dosage. Venous blood was collected on an empty stomach in the early morning of the next day after double antibody drug therapy in hospital, and routine examination results were recorded, including routine blood test, coagulation function, biochemical items, blood lipid items, glycosylated hemoglobin, and oral glucose tolerance test.

#### 2.2.3. Detection of Thromboelastogram and Determination of Related Parameters

Seven days after patients took double anticoagulant medicines, venous blood was collected on an empty stomach in the next morning and injected into sodium citrate anticoagulant tube 1 and heparin anticoagulant tube 2, respectively. Afterwards, we put the test cup into the cup slot of the analyzer and input the sample data in the data column of the TEG operation interface; citric acid-kaolin samples were tested to obtain the maximum amplitude of MA_THROMBIN_ (MA value of thrombin), MA_FIBRIN_ (MA value of fibrin), and other TEG parameters. Samples activated by A (activator F), ADP (adenosine diphosphate), and AA (arachidonic acid) were examined. AA and ADP inhibition rates were gained by TEG software analysis.

AA%: the platelet inhibition rate produced by the AA pathway, and ADP%: the platelet inhibition rate produced by the ADP pathway.

AA% ≤ 50% represents aspirin low reactivity (resistance) [13], and 50% represents aspirin high reactivity; ADP% ≤ 30% means the low reactivity (resistance) of clopidogrel [14], and 30% means the high reactivity of clopidogrel.

The interpretation of relevant parameters of TEG is as follows [15]:

1. *R* time: reaction time refers to the time spent on the formation of the first thrombus; it embodies the function of coagulation factor; the reference range is 5–10 min
2. *K* time: it is the time from the reaction time until the thrombus amplitude reaches 20 mm; it embodies the fibrinogen function; the reference range is 1–3 min
3. Parameters: thrombus formation speed; it also reflects the function of fibrinogen; the reference range is 53–72 deg
4. MA value: maximum amplitude, mainly reflecting platelet activity and function; the reference value range is 50–70 mm
5. Coagulation composite index: it represents the overall coagulation state, predicting bleeding and ischemia (−3 is low coagulation, and +3 is high coagulation)
6. *G*: blood clot strength, a parameter reflecting thrombus hardness
7. *E*: elastic constant, a parameter reflecting thrombus hardness
8. TPI: platelet dynamic index, which reflects the parameters of blood coagulation function; 6TPI15 is in the normal coagulation state
9. A: instantaneous amplitude
10. A30: the amplitude at 30 min
11. CL30: the percentage of thrombus left after dissolution in half an hour (CL3092.5% indicates hyperfibrinolysis)
12. LY30: the rate of thrombus reduction in half an hour, reflecting fibrinolytic function; LY307.5% indicates hyperfibrinolysis
13. EPL: percentage of thrombolysis, representing fibrinolytic function; the reference value is 0–15%

### 2.3. Statistical Analysis

The data were assessed by SPSS25.0 statistical software. Those in accordance with normal distribution were expressed by mean ± standard deviation (±*S*). The nonnormal distribution is represented by [*M* (*P*25, *P*75)]. The comparison between the two groups was made by an independent-sample *T* test, and that among multiple groups was made by variance analysis. The counting data were expressed in frequency and percentage (%). The chi-square test was used for comparison between groups of two classified variables, and logistic regression was applied in multivariate analysis. *P* < 0.05 denotes that the difference is statistically significant.

## 3. Result Analysis

### 3.1. Analysis of Patient Data

#### 3.1.1. Basic Pathological Data of Patients

Totally 118 CHD patients at the altitude of 2125–4272 m were included in this study, aged 38–84 years, including 81 males (68.64%), 37 females (31.36%), 42 Tibetans (35.59%), and 76 Han (64.41%). The characteristics of clinical diseases and hematological indicators are shown in Figure 1 and Table 1. The platelet function and coagulation-fibrinolysis function were tested by TEG, and MA_THROMBI_, MA_ADP_, and MA_AA_ were all higher than the reference range, as shown in Table 2.

### 3.2. Analysis of Risk Factors of Drug Resistance

#### 3.2.1. Comparison between ACS and CCS Groups

There was no dramatic difference in age, gender, BMI, oxygen saturation, TG, GFR, and history of diabetes and hypertension between both the groups (*P* < 0.05) (Figure 2). PLT and FIB in the ACS group were higher than those in the CCS group, and the difference was statistically significant (*P* < 0.05). In addition, MA_THROMBIN_, MA_FIBRIN_, E, A, A30, and coagulation composite index were also higher than those in the CCS group, a with statistically significant difference (*P* < 0.05), as shown in Tables 3 and 4.

#### 3.2.2. Analysis of Risk Factors of Drug Resistance

*(1) Incidence of Drug Resistance*. Among 118 CHD patients, 82 cases (69.49%) had drug resistance and 36 cases (32.53%) were drug-susceptible. The incidence of AR was 56.78% (67 cases), among which 17 cases (14.41%) were AR alone; there were 65 cases of CR, and the incidence rate was 55.08%, of which 16 cases (12.71%) were CR alone, as shown in Table 3.

*(2) Univariate Analysis of Risk Factors of Drug Resistance*. Compared with the drug-sensitive group, there were remarkable differences in age, gender, HbA1c, MAO, GFR, FBG, application of proton pump inhibitors, and diabetes (*P* < 0.05), as shown in Figure 3(b).

*(3) Logistic Regression Analysis of Risk Factors of Drug Resistance*. Univariate analysis of variance demonstrated that there were obvious differences in age, gender, HbA1c, MAO, GFR, FBG, application of proton pump inhibitors, and diabetes (*P* < 0.05). With the abovementioned factors as independent variables and drug resistance as dependent variables, a binary logistic regression analysis was performed, as shown in Table 5. Age is an independent risk factor for drug resistance, and the risk of drug resistance increases by 18.6% for every one year of age increase; HbA1c is an independent risk factor of drug resistance, and the risk of drug resistance increases by 10.125 times for every 1% increase of HbA1c; the increase of FBG is an independent risk factor of drug resistance, and the risk of drug resistance increases 1.108 times for every 1 mmol/L increase of FBG; diabetes is an independent risk factor for drug resistance, and the risk of drug resistance in diabetic patients is 9.945 times that in those with diabetes, as shown in Figure 4.

## 4. Discussion

With the acceleration of globalization and population aging, CHD, as one of the major diseases threatening the health of the whole people, has become the main cause of death of cardiovascular and cerebrovascular diseases [16]. As the secondary prevention of CCS, antiplatelet therapy has made great progress in reducing MACE [17]. Nevertheless, with the wide application of antiplatelet therapy, aspirin resistance and clopidogrel resistance have been paid more and more attention by scholars at home and abroad because of their influence on efficacy. This study aims to reveal the platelet function and coagulation-fibrinolysis function of CHD patients in the Qinghai area and then to understand the difference of abovementioned functions between two kinds of patients; it clarifies the incidence of aspirin resistance and clopidogrel resistance in Qinghai and the related biochemical factors affecting the occurrence of aspirin and clopidogrel resistance, so as to optimize the antithrombotic treatment scheme for CHD patients at high altitude and provide basis for individualized study of antithrombotic treatment.

The MA_THROMBIN_ value of platelet function in 118 CHD patients at high altitude was higher than the reference range, suggesting that platelet activity of CHD at high altitude was enhanced. Darlene et al. have proposed that high altitude is a potential risk factor for thrombosis by studying the incidence of thromboembolic events at high altitude of 3000–8000 m [18]. Alistair et al. [19] have measured the blood changes of 63 healthy volunteers from plain areas who come to high altitude regions first (5200 m), so as to explore the influence of high-altitude hypoxia on the number and function of platelets and then found the regional differences of patients and the differences of platelet activity. In this study, the incidence of AR and CR was 56.78% and 55.08%, which was higher than that of other plain areas in China, with the same time, detection method, and judgment standard, such as Shanghai [20] (AR16.49% and CR3.43%), Guangdong [21] (AR13.00% and CR10.00%), and Beijing (AR14.92% and CR5.66), with a statistically significant difference (*P* < 0.05) [22]. Moreover, research has shown that [23] hypoxia at high altitude has a remarkable impact on the activities and behaviors of organisms, which may change the expression and activity of drug metabolism enzymes. In aspirin and clopidogrel treatment of antiplatelet reaction, high incidence of AR and CR in the high-altitude area may be relevant to the genetic background of the population. At last, in the study of the factors of drug resistance, it is found that there is a direct relationship between the occurrence of drug resistance and the increase of age, diabetes, and blood glucose. Patricia [24] observed 325 CHD patients and found that age is a risk factor of AR. Due to the lack of representation of the elderly in clinical trials, the studies on pharmacokinetics (PK) and pharmacodynamics (PD) in the elderly are not yet mature, and the safety and effectiveness of drugs are in doubt. Paven investigated 116 patients with type 2 diabetes [25] and found that AR was correlated with the duration of diabetes and higher fasting blood glucose (FBS) level. Hakan et al. put forward that AR in type 2 diabetic patients [26] might be tied to the increase of platelet aggregation caused by the rise of acute phase reactive protein in plasma. The abovementioned related studies indicate that the increase of FBS caused by age and diabetes will increase the risk of clinical medication.

Limitations of the study: this study analyzed the reactivity and influencing factors of aspirin and clopidogrel in CHD patients at high altitude, but all the samples came from the same hospital, which may lead to selection bias. In the meantime, the study noted that the incidence of aspirin and clopidogrel resistance in CHD patients at high altitude was higher than that in plain areas, but the differences caused by the genetic background of the population were not further explored. Hence, the study still needs further discussion.

## Figures and Tables

**Figure 1:** Summary chart of patients' basic situation.

**Figure 2:** Comparison between ACS and CCS groups.

**Figure 3:** Comparison of occurrence ratio and counting data of drug resistance.

**Figure 4:** Analysis of pathological factors of drug resistance.

**Table 1:** Description of hematological indexes of enrolled cases.

Projects	±*S*/*M*(*P*_25_, *P*_75_)
Routine blood test	
RBC (10^12^/L)	4.850.78
HBG (g/L)	149.0424.16
MCV (fL)	93.417.86
MCHC (pg)	30.056.21
PLT (10^9^/L)	183.4661.64
PCT (%)	0.200.05
PDW (%)	15.103.45
MPV (fL)	11.521.32
P-LCR (%)	37.5510.38

Coagulation function	
PT (sec)	12.00 (11.55, 13.03)
APTT (sec)	28.314.67
FIB (g/L)	2.80 (2.37, 3.54)
D-D (g/mL)	1.05 (0.81, 2.45)
FDP (g/mL)	2.66 (2.03, 4.71)

*Note.* RBC = red blood cell, HBG = hemoglobin, MCV = mean corpuscular volume, MCHC = mean corpuscular hemoglobin concentration, PLT = platelet, PCT = plateletcrit, PDW = platelet distribution width, MPV = mean platelet volume, P-LCR = platelet-larger cell ratio, PT = prothrombin time, APTT = activated partial thromboplastin time, FIB = fibrinogen, D-D = D-dimer, FDP = fibrin degradation products.

**Table 2:** Description of main parameters of TEG in patients.

Projects	Parameter value	Reference value
R [min *M* (*P*_25_, *P*_75_)]	6.4 (5.2, 7.2)	5–10
K [min *M* (*P*_25_, *P*_75_)]	2.1 (1.6, 2.9)	1–3
[deg *M* (*P*_25_, *P*_75_)]	62.45 (52.10, 68.92)	53–72
MA_THROMBI_ (mm, *x* ± *S*)	66.366.73	50–70
MA_FIBRIN_ [mm, *M*(*P*_25_, *P*_75_)]	12.35 (9.07, 15.12)	—
MA_ADP_ (mm, *x* ± *S*)	48.6513.95	31–47
MA_AA_ (mm, *x* ± *S*)	42.1510.03	31–47
Coagulation composite index [*M* (*P*_25_, *P*_75_)]	1.60 (−0.53, 3.03)	−3–3

**Table 3:** Comparison of platelet and coagulation function parameters between ACS and CCS groups (±*S*).

Projects	ACS group (*n* = 66)	CCS group (*n* = 52)	*t*/*z*	*P*
Platelet parameters				
PLT (10^9^/L)	198.7273.16	170.0054.68	2.358	0.020
MPV (fL)	11.531.45	11.751.27	0.864	0.390
P-LCR (%)	35.6712.29	37.029.85	1.601	0.112
PCT (%)	0.21 ± 0.15	0.19 ± 0.16	0.698	0.486
PDW (%)	14.00 ± 2.89	14.50 ± 3.21	0.889	0.376

Coagulation function				
APTT (sec)	28.745.14	27.763.97	1.134	0.259
FIB (g/L)	3.631.45	3.050.96	2.486	0.014
TT (sec)	18.454.00	18.091.49	0.616	0.539

**Table 4:** Comparison of TEG parameters between ACS and CCS groups [±*S*].

TEG parameters	ACS group (*n* = 66)	CCS group (*n* = 52)	*t*/*z*	*P*
*R* (min)	6.20 ± 1.98	6.50 ± 1.20	0.962	0.338
*K* (min)	2.30 ± 1.12	2.25 ± 1.08	0.245	0.807
(deg)	62.19 ± 19.85	64.92 ± 25.36	0.656	0.513
MA_THROMBIN_ (mm)	67.876.60	64.406.43	2.957	0.004
MA_FIBRIN_ (mm)	13.207.8	10.204.5	2.181	0.031
MA_ADP_ (mm)	48.7113.36	48.5714.79	0.054	0.957
MA_AA_ (mm)	41.2113.10	38.7714.98	0.977	0.330
Coagulation composite index	2.310.82	0.490.93	11.281	0.001
*G*	101.0565.23	87.0056.38	1.232	0.220
*E*	206.7559.89	173.6969.35	2.776	0.006
TPI	45.8332.16	41.6629.68	0.723	0.471
A (mm)	66.816.92	62.2910.53	2.899	0.004
A30 (mm)	66.417.28	62.678.95	2.586	0.011

*Note.* TPI = thrombodynamic potential index.

**Table 5:** Logistic regression analysis of risk factors of drug resistance.

Independent variable	*B*	S. E	Wald	*P*	OR, 95% CI
Woman	1.822	1.409	1.673	0.196	6.186 (0.319∼97.857)
Age	0.170	0.051	11.289	0.001	1.186 (1.074∼1.309)
HbA1c	3.816	1.217	9.829	0.002	11.125 (2.253∼87.624)
FBG	0.746	0.338	4.878	0.027	2.1089 (1.088∼4.087)
MAO	0.120	0.155	0.606	0.436	1.128 (0.833∼1.528)
GFR	−0.006	0.021	0.067	0.795	0.994 (0.954∼1.037)
PPIs	1.465	1.133	1.673	0.196	4.328 (0.470∼39.851)
Diabetes	2.297	0.847	7.350	0.007	9.945 (1.890∼52.339)

## Data Availability

The primary data to support the results of this study are available at reasonable request to the corresponding author.
